# Postoperative Examination of Laryngeal Malignant Tumor Based on Narrowband Imaging Resolution Enhancement Technology

**DOI:** 10.1155/2022/7762622

**Published:** 2022-05-28

**Authors:** Neng Yang, Chenchen Zhao, Fenfen Lin, Jiaojiao Wu, Ben Liu

**Affiliations:** ^1^ENT Department, Taizhou Hospital of Zhejiang Province Affiliated to Wenzhou Medical University, Zhejiang, Taizhou 317000, China; ^2^Department of Operating Room, Taizhou Hospital of Zhejiang Province Affiliated to Wenzhou Medical University, Zhejiang, Taizhou 317000, China

## Abstract

The application of endoscopic imaging in the biopsy of malignant laryngeal lesions is one of the current research hotspots in the medical field. Based on the narrowband imaging resolution enhancement technology, a model for postoperative examination of laryngeal malignant tumor was constructed in this paper. The article calculated the biopsy detection rate of malignant lesions and the correct biopsy detection rate of the two groups and made a statistical comparison. In the NBI mode group, the mucosal morphology and superficial mucosal microvascular morphology of the same lesion under two different modes of white light and NBI were compared, which solved the problem of data processing of cases. During the case comparison process, patients who needed biopsies to be sent for pathology were selected for inclusion in the study and were randomly divided into two groups. The coincidence rate of EUS combined with NBI diagnosis was significantly higher than that of ordinary white light gastroscopy (47.92%), and the difference was statistically significant (*P*=0.000 < 0.05). The experimental results compared the accuracy of the normal white light mode and the NBI mode to diagnose the nature of the lesions: according to the Kudo classification criteria, 23 cases of tumor lesions were to be diagnosed in the normal white light mode, with an accuracy rate of 69.70%, and the NBI mode was to be used to diagnose tumors. There were 81 cases of sexual lesions, with an accuracy rate of 93.94%. The NBI mode was more accurate in diagnosing the nature of the lesions under the Kudo classification standard (*P* < 0.05). In 64 cases, the accuracy rate was 63.63%. Under the NBI mode, 29 cases of tumor lesions were proposed to be diagnosed, and the accuracy rate was 87.88% to promote the application of NBI endoscopy in the biopsy of malignant laryngeal lesions.

## 1. Introduction

The basic principle of narrowband imaging technology is to narrow the white light wavelength of the xenon lamp into narrowband light waves of blue (wavelength 415 nm), green (wavelength 540 nm), and red (wavelength 600 nm) through special filters, mainly emphasizing blue light [1]. This narrowband light wave dominated by blue light has weak penetrating power and shallow irradiation depth and can only reach the surface of the tissue, thereby increasing the contrast and clarity of the mucosa, so it can clearly display the mucosal surface structure and gland duct opening shape [2–5]. In addition, due to the strong absorption of blue light by the optical characteristics of hemoglobin, NBI can also clearly display the submucosal microvascular morphology. The image provided by optical enhancement technology emphasizes the morphology and surface structure of mucosal blood vessels and enhances the visibility of blood vessels and other structures on the mucosal surface, which is conducive to the detection of lesions and enables it to obtain a visual effect similar to that of chemical staining under endoscopy [6–8].

The histopathological type of most malignant laryngeal lesions is squamous cell carcinoma. Although the etiology of laryngeal carcinoma (LC) is not fully understood, it is generally believed that it may be related to air pollution, smoking, alcohol consumption, human papillomavirus infection and sex hormones [9–12]. With the development of bad habits such as smoking and drinking, and the aggravation of environmental pollution such as the emission of a large amount of dust and exhaust gas, the combined effect of various carcinogenic factors has caused the incidence of laryngeal cancer to increase year by year, becoming the second largest with high incidence of cancer of the respiratory tract. Not only that, but some benign lesions such as vocal cord leukoplakia and laryngeal papilloma are easily transformed into laryngeal cancer, which increases the potential incidence of laryngeal cancer [13–16]. The clinical symptoms of laryngeal cancer vary according to the location of the lesions: glottic laryngeal cancer can have symptoms such as hoarseness in the early stage of the onset, while lesions in other parts often have no obvious symptoms or atypical symptoms in the early stage, even if the tumor has developed to a certain extent. The degree of symptoms is only mild or nonspecific, mostly manifested as throat discomfort, pain, or foreign body sensation, etc. Only in the advanced stage of laryngeal cancer will obvious dyspnea, swallowing obstruction, coughing and hemoptysis, blood in sputum, or neck mass such as cervical lymphadenopathy appear. Therefore, timely and accurate detection of malignant laryngeal lesions will help clinicians to formulate correct diagnosis and treatment plans in the early stage of the lesions, effectively prevent malignant lesions from continuing to invade surrounding tissues, and avoid the expansion of surgical scope and the loss of voice function of patients due to delayed diagnosis case [17–19].

At present, the main clinical examination methods are CT, MRI, endoscopy, laryngeal cancer marker thymidine kinase, squamous cell carcinoma-related antigen, etc., but the latter two have a longer diagnostic cycle, and the former three are commonly used. It should be noted that the diagnosis rate of cancerous lesions can be significantly improved by repeatedly cleaning the lesions with normal saline and then switching to NBI mode for observation and targeted biopsy of the suspected lesions. Imaging examination can play a very important role in judging the degree of lesion invasion and cervical lymph node metastasis, but it has limited ability for those early cancers that only occur in the superficial mucosa, and only endoscopy can directly detect lesions on the mucosal surface. It can identify and take a biopsy under direct vision, obtain histological evidence, and diagnose laryngeal diseases accurately and in a timely manner. The diagnostic accuracy of traditional endoscopy for laryngeal cancer depends largely on the clinical experience of ENT specialists and can only be identified when the lesions have obvious morphological changes. By spraying a living dye on the mucosal surface, the color difference between diseased tissue and normal tissue can be distinguished, thereby enhancing the ability of visual recognition under the microscope and improving the detection rate of lesions.

## 2. Related Work

Narrowband imaging technology (narrowband imaging NBI) uses a filter to filter out the broadband spectrum in the red, blue, and green light waves emitted by the endoscope light source, leaving only the blue, green, and red narrowband light waves with wavelengths of 415 nm, 540 nm, and 600 nm. It increases the contrast and clarity of mucosal epithelial and submucosal vascular patterns and improves the observation details of mucosal surface microstructure and microvascular morphology, thereby improving the accuracy of endoscopic diagnosis. In recent years, some reported that the “light blue crest” on the epithelial surface of the laryngeal mucosa is a manifestation of NBI combined with magnifying laryngoscopy that is closely related to laryngeal mucosal epithelial metaplasia.

Raj et al. [20] believed that NBI was better than traditional endoscopy for depression contours and better for mucosal vascular network and lesion tone than traditional endoscopy and had a sensitivity of 100% in distinguishing neoplastic and nonneoplastic lesions. The specificity was 75%, superior to conventional endoscopy (sensitivity 83%, specificity 44%) and similar to results of chromoendoscopy. Lee et al. [21] and others reported using NBI combined with magnifying endoscopy to observe 11 patients with BE. The results showed that the sensitivity and specificity of ordinary endoscopy in detecting SIM were 24% and 67%, respectively; NBI was 56% and 56%, respectively. 95%; chromoendoscopy was 55% and 100%. It can be seen that NBI is significantly better than ordinary endoscopy and its results are similar to the results of chromoendoscopy. According to Tirelli et al. [22], the clinical application in recent years shows that NBI is significantly better than ordinary endoscopy in finding early mucosal lesions and clear lesions and can be used to evaluate the scope of precancerous lesions and early laryngeal cancer in a retrospective study. Its sensitivity for diagnosing laryngeal cancer is 96.4%, which is significantly better than traditional endoscopy, and the results observed by endoscopists with different experience levels under fluorescence endoscopy have good consistency, so the accuracy of fluorescence endoscopy is less dependent on the diagnosis and experience of endoscopists. However, fluoroscopic endoscopy has certain limitations: the specificity is poor, only 49.1%, especially when combined with laryngeal ulcers, it has a higher false positive rate, and although the sensitivity is worse than that of traditional endoscopy, it is not as good as narrowband imaging endoscopy.

Studies have shown that NBI magnifying endoscopy can improve the diagnostic accuracy of neoplastic lesions according to the changes of surface structure and microvessels of gastrointestinal mucosa. Nata's et al. [23] study believed that ultrasound laryngoscopy could diagnose the depth of tumor invasion, tissue metastasis, and lymph node metastasis with an accuracy of 80% and could guide endoscopic treatment of early laryngeal cancer. Maeda et al. [24] pointed out that, combined with fine needle aspiration biopsy, endoscopic ultrasonography can well detect EGC and perform preoperative staging and accurately predict the feasibility of endoscopic treatment, so that some patients may suffer from it. Avoiding laryngectomy is especially important for older adults who have other complications that are not suitable for surgery. However, endoscopic ultrasonography is expensive, requires high theoretical and operational skills for endoscopists, and has different imaging quality, which limits the popularization of endoscopic ultrasonography. The researchers used confocal laser endomicroscopy for clinical observation of gastrointestinal mucosa, and the obtained real-time microscopic images were also in good agreement with traditional histopathological images, so they believed that confocal laser endomicroscopy can display the tissue structure of digestive tract mucosa and submucosa and make instant diagnosis of laryngeal cancer and precancerous lesions in vivo. However, confocal laser endoscopy equipment is expensive and the clinical application time is short. Currently, research work is only carried out in a few large hospitals in China. There are still many problems to be solved urgently in terms of endoscopic image quality and diagnostic technical standards [25, 26].

## 3. Case Examination of Narrowband Imaging Resolution Enhancement Technology

### 3.1. Evaluation of Narrowband Imaging Preference

Narrowband imaging can increase the contrast and clarity of mucosal epithelium and submucosal vascular patterns and improve the observation details of mucosal surface microstructure and microvascular morphology, thereby improving the accuracy of endoscopic diagnosis. The relevant data of the included studies were collected independently by two authors. The data to be collected and extracted include the first author of the included studies, the year of publication, the country, the number of cases included in each group, the sex ratio, the average age, the time to withdraw from the mirror, and the detection of polyps. For the same data, if the two authors disagree, they will be resolved through discussion.

(1) $$\begin{array}{c} Y\left(x\left(i,j\right),t\left(i,j\right)\right)=\frac{\text{delta}\left(di-dj\right)}{\text{delta}\left(di+di\right)}-\frac{\Delta t\left(i,j\right)}{x\left(i,j\right)}. \end{array}$$

In this paper, the Cochrane risk bias assessment tool was mainly used, and the selection bias, implementation bias, measurement bias, and followup bias of the included studies were assessed by two authors respectively. Similarly, if the two parties disagree, they should be resolved through discussion. If the discussion still cannot be determined, a third party will be invited to intervene and vote to decide the disagreement.

Referring to the Sano CP classification and Kudo's pit pattern classification, all the lesions found were subjected to pit pattern classification in the magnification mode of Figure 1, and CP classification was performed in the NBI magnification mode. The pathological results were compared, and the tumor or nonneoplastic lesions were diagnosed according to the typing results. At the same time, the results were compared with the pathological results. Therefore, polypoid lesions should be routinely biopsied to clarify their pathological types and guide endoscopic followup and treatment. By EUS combined with NBI, it was found that the gastric pits with noncancerous lesions, low-grade intraepithelial neoplasia, or intestinal metaplasia were mostly of type A, type B, and type C, which were regular and symmetrical. The diagnostic accuracy was 91.8% (134/146), 92.6%, and 90.4%, respectively; the coincidence rate, sensitivity, and specificity of CP classification in the diagnosis of large laryngeal neoplastic lesions under NBI magnification mode were 90, 4% (132/146), 94.6%, and 82.7%, respectively. There was no statistically significant difference between the two (gizzard O.05), but both were higher than those of conventional endoscopy (79.4%, 74.6%, and 84.4% (*P* < 0.05)).

### 3.2. Pathological Analysis of Laryngeal Malignant Tumors

In the pathology of 67 cases of laryngeal malignant tumors, 18 cases were of homogeneous particle type, 24 cases of mixed nodule type, 23 cases of flat and raised type, and 2 cases of pseudodepressed type. The average age of LST patients was 62.00 + 13.69 years, and the average diameter was 24.40 ± 15.72 mm. There were 31 (46.3%) male patients and 36 (53.7%) female patients. The lesions are mainly located in the straight throat, accounting for 38.8% (26/67). The average age of patients with homogeneous particles in Table 1 is 57.83 ± 17.22 years, and the average diameter is 23.117 ± 13.46 mm. There are 5 male patients and 13 female patients. The lesions mainly occur in the straight larynx, accounting for 38.9% (7/18).

The patients with mixed nodules had an average age of 65.67 + 10.19 years and an average diameter of 33.08 + 20.13 mm, including 11 (45.8%) male patients and 13 (54.2%) female patients. The lesions were mainly located in the straight larynx, accounting for 58.3% (14/24). The average age of the patients with flat and elevated type was 61.04 + 13.37 years, and the average diameter was 16.74 ± 5.41 mm, including 14 (60.9%) male patients and 9 (39.1%) female patients.

(2) $$\begin{array}{c} \forall x\left(i,j\right)\in X\left\{\begin{array}{c} i=1,2,3,,,n\\ j=1,2,3,\ldots ,i-1 \end{array}\right),\;\exists !x\left(i,j\right)=1\frac{n!}{r!\left(n-r\right)!}. \end{array}$$

The lesions mainly occurred in the descending larynx, accounting for 26.1% (6/23). The average age of the pseudodepressed patients was 66.5 ± 17.68 years, and the average diameter was 20 ± 7.07 mm, including 1 (50%) male patient and 1 (50%) female patient. There was no significant difference between the different endoscopic types of LST and the age, gender, lesion diameter, and disease site of the patients (*P* > 0.05).

### 3.3. Resolution Digital Enhancement

SPSS 20.0 statistical software was used to analyze the resolution digital data, the normal distribution data was described by mean ± standard deviation, the measurement data were compared between two groups by *t* test, and the enumeration data were compared by ×2 test or Fisher's exact probability method, described in *P*. About 35% of LDT-G had tubular villiform structures, but no villiform structures were found in flat-raised LST lesions, which may be related to the higher malignant potential of the latter. EUS mode was switched to carefully observe the layers of the digestive tract wall at the lesion site and the relationship between the lesion and each hierarchical structure. After obtaining clear ultrasound images, the ultrasound images were frozen and saved, and the nature of the lesion was determined according to the lesion location, shape, size, boundary, origin level, ultrasonic echo characteristics, and tumor invasion.

(3) $$\begin{array}{c} \left\{\begin{array}{c} 1-\text{if}\left(u\left(n\right),v\left(n\right)\right)<1,\\ 1+\text{if}\left(u\left(n\right),v\left(n\right)\right)>0. \end{array}\right) \end{array}$$

Some scholars found that, after statistics of 92 LST cases, LST-F did not have a tubular villi structure, but LST-G showed a tubular villi structure and accounted for 28.3%. Different types of LST have different malignant potential, but their malignant potential has little relationship with tumor diameter. The malignant potential of LST-G is higher than that of polypoid lesions, but lower than that of LST-F.

Among physicians with similar ADRs, the missed diagnosis rates were not the same. The average number of adenomas detected by the participants can well distinguish the endoscopists who blindly pursue high ADR from the endoscopists who make careful inspections, which is another important indicator for evaluating the quality of endoscopy in Figure 2. We analyzed the mean number of adenomas detected, the mean number of polyps detected, and the mean number of flat adenomas detected and found that there was no statistical difference in the mean number of adenomas detected and the mean number of polyps detected. The mean number of flat adenomas detected in NBI was higher than that in WLC, with a statistically significant difference; this conclusion is consistent with ADR. Therefore, from the ADR and the mean number of adenoma detections in the participants to jointly evaluate NBI and WLC, it can be concluded that NBI is not superior to WLC in the detection of adenomas and polyps, but NBI can better detect flattened than WLC adenoma.

### 3.4. Clustering of Case Lesion Biopsy Samples

The main complaint of the biopsy sample of the lesion was throat discomfort or foreign body sensation, with or without hoarseness, and blood in the sputum. The larynx mass was found by electronic nasolaryngoscopy screening, and malignant lesions were suspected. Biopsy was required for pathological examination in 113 cases. All patients were divided into 58 cases in the white light mode group and 55 cases in the NBI mode group according to the single-day and double-day randomization method (the patients who visited the clinic on a single day were included in the white light mode group, and those who visited the clinic on two days were included in the NBI mode group).

(4) $$\begin{array}{c} \frac{\text{thenwer}\left(t+\text{delta}\left(t\right)\right)}{u\left(n,t\right)}-\frac{\text{derta}\left(t\right)}{\text{derta}\left(n\right)}=1. \end{array}$$

In the white light mode group, the laryngeal examination was performed in the white light mode, and after leaving the image data, a biopsy of the laryngeal lesion was taken and sent for pathological examination. Laryngeal lesions were biopsied and sent for pathological examination. Based on ordinary white light electronic endoscopy, NBI endoscopy filters white light to display only narrowband light waves, so as to significantly enhance the contrast and clarity of mucosal layer and submucosal blood vessels and display the fine structures of mucosal surface more clearly.

(5) $$\begin{array}{c} u\left(i,i+1\right)-v\left(i,i+j\right)>v\left(i,i+1\right)-u\left(i,i+j\right)+\text{derta}\left(i,j\right). \end{array}$$

Both groups of patients underwent corresponding surgical operations according to the histopathological results of biopsy tissue, and the surgically resected tissue was sent for pathological examination, and histopathological results were used as the gold standard. The biopsy detection rate and correct biopsy detection rate of malignant lesions in the two groups were calculated and compared statistically. In the NBI mode group in Figure 3, the mucosal morphology and the superficial mucosal microvascular morphology of the same lesion under two different modes of white light and NBI were compared.

The capillary thickening of the adenoma lesions is relatively uniform, and in the NBI mode, it appears as a regular network of brown capillaries surrounding the opening of the gland, and the structure of the opening of the gland is also regular. On the other hand, the capillaries on the surface of adenocarcinoma are unevenly thickened, unevenly arranged, and unevenly distributed. According to the Sano classification, NBI technology combined with magnifying endoscopy technology has an accuracy rate of 95.5% in identifying adenoma and adenocarcinoma. The pathological biopsy tissue or postoperative gross specimen should be examined and diagnosed by experienced pathologists, with the pathological histological diagnosis as the standard.

## 4. Construction of Postoperative Examination Model for Laryngeal Malignant Tumor Based on Narrowband Imaging Resolution Enhancement Technology

### 4.1. Narrowband Imaging Resolution Data Processing

After analysis of the narrowband imaging resolution data, the results suggested that there was no statistical difference between NBI and WLC (22.7% vs. 20.7%, *P*=0.17, RR 1.12; 95% CI 0.96–1.30) (*I*^2^ = 38%), there is mild heterogeneity, and the heterogeneity analysis was carried out by the exclusion method one by one. The results before and after exclusion were consistent, indicating that the results of this analysis were reliable, suggesting that NB cannot reduce the missed diagnosis rate of adenomas compared with WLC. Among the 67 patients with laterally developing tumors, tubular adenoma was the main pathological type, accounting for 40.3% (27/67).

(6) $$\begin{array}{c} \frac{d\left(u\left(n\right),v\left(n\right)\right)-p\left(u\left(n\right),v\left(n\right)\right)}{du\left(n\right)-dv\left(n\right)}-\frac{at-bt^{2}}{dt}-c=0. \end{array}$$

Endoscopic typing and pathological typing were compared and analyzed, and Fisher's exact probability analysis showed that there was a significant difference between microscopic typing and pathological typing (*P* < 0.01). The endoscopic types of 6 cases of intramucosal carcinoma were all mixed nodule type, 2 cases of 3 cases of submucosal carcinoma were found in mixed nodule type, and 1 case was found in flat-raised type, suggesting mixed nodular and flat-raised lesions.

(7) dun,vndun,vn−1+1⟶datat−bt^2−c.

Cancer rate is high. When endoscopy is diagnosed as mixed nodule type and flat-raised type, it needs to be combined with ME. NBI carefully observes the microstructure of the lesion surface and is alert to the possibility of growing into a cancer.

ADR can be achieved with HD-NBI compared to HD-WLC regardless of the experience of the endoscopist. NBI technology is currently the most commonly used electronic chromoendoscopy technology, which has been widely used in the monitoring of adenomas because of its simple and fast operation and the ability to switch the field of view with one button. In order to further clarify whether NBI is conducive to improving ADR, we included 16 high-quality RCTs in Figure 4 for a systematic meta-analysis, with a total of 7401 patients included, which can more effectively answer the statistical question of whether NBI can improve ADR. Unfortunately, NBI does not improve ADR compared to WLC. When we analyzed the PDR, the results showed that there was still no clear benefit. Mesenchymal tumors were characterized by uniform hypoechoic mass originating from the musculature propria. The mucosal layer and mucosal musculature of mesenchymal tumors with ulcerated surface were characterized by local defects of varying degrees. Lipoma is characterized by homogeneous hyperechoic mass originating in the submucosa.

### 4.2. Calculation of Postoperative Recovery Rate for Laryngeal Lesions

Standard single-man operation for laryngeal lesions, from entering the endoscope to the backward endoscope for observation, and using the ME-NBI mode to observe the lesions and save the images after white light endoscopy finds suspicious lesions. Careful observation of the Pit pattern classification and Sano capillary classification of the LST gland opening under endoscopy, combined with other morphological characteristics of the lesions, such as size, location, endoscopic morphological classification, and postoperative pathological tissue classification, were used to discuss ME diagnostic value of NBI for LST. All endoscopic pictures were evaluated by more than 2 experienced endoscopists to evaluate the mucosal surface microstructure and submucosal capillary classification on the lesion surface.

(8) $$\begin{array}{c} \frac{1-u\left(i,j\right)}{\text{epwsideu}\left(\left(i,j\right)+u\left(0\right)+1\right)}-\frac{\Delta \left(1-u\left(i,j\right)\right)}{\Delta \text{epwside}\left(u\left(i,j\right)+u\left(0\right)+1\right)}=\frac{1}{\Delta \left(1-u\left(i,j\right)\right)}. \end{array}$$

In our study, we found that when NBI-ME was used to observe laryngeal mucosal lesions, the size and shape of the laryngeal pits at the lesions were diverse, and the Sakaki classification with relatively fine typing was used, and the detailed classification of the laryngeal pits was more maneuverable; some lesions often have two or more areas of laryngeal fovea morphological changes. The correlation between the obtained pathological results and laryngeal fovea morphological changes is not easy to determine.

(9) $$\begin{array}{c} u\left(i,j\right)x\left(i,j-i\right)\left(t,t-\text{derta}\left(t\right)\right)=\frac{u\left(i-1,j-1\right)}{d\left(t,t-\text{derta}\left(t\right)\right)}. \end{array}$$

The Tanaka classification, which is relatively broad, is used to study the laryngeal fovea morphology. The correlation between changes and pathological results was more maneuverable. The key of NBI-ME in the diagnosis of early laryngeal cancer is clear imaging. The fine structure of normal laryngeal mucosa is different in different parts of the larynx, and its morphological distribution is regular.

Using NBI and HD-WLC to compare and analyze their PDR, the results in Figure 5 were also not statistically different (43.7% vs. 41.6%, *P*=0.32, RR 1.09; 95% CI 0.92–1.30, *I*^2^ = 77%). If *I*^2^ > 75%, it indicates high heterogeneity, and the included studies were excluded one by one for heterogeneity analysis; the results before and after exclusion were consistent, and the results of this analysis were reliable, suggesting that NBI cannot improve PDR compared with HD-WLC. At the same time, the heterogeneity in this subgroup may be the source of the heterogeneity between the NBI and WLC comparison groups.

### 4.3. Comparison of Histological Results of Laryngeal Malignant Tumors

From the patients who visited the otolaryngology head and neck surgery, the main complaints were throat discomfort, pain or foreign body sensation, with or without hoarseness, blood in the sputum, and a laryngeal mass found by electronic nasolaryngoscopy screening, and malignant lesions were suspected, and cases requiring biopsy and sent for pathology were included in the study.

(10) $$\begin{array}{c} \sqrt{u\left(i,j\right)}-\sqrt{\left(t,t-\text{derta}\left(t\right)\right)}=\sqrt{x\left(i,j-i\right)}-\sqrt{u\left(i-1,j-1\right)}. \end{array}$$

Exclusion criteria were as followed: (1) allergy or hypersensitivity to lidocaine in the past, (2) uncontrolled dyspnea, uncontrolled bleeding disease, and severe cardiovascular disease, (3) intolerance to endoscopy, (4) those who cannot understand the relevant conditions, the purpose of endoscopy, risks, and precautions, or those who refuse to sign the informed consent, and (5) those who have undergone surgery for laryngeal cancer or are undergoing radiotherapy and chemotherapy. A total of 113 cases were collected, including 95 males and 18 females, aged between 42 and 80 years, with an average age of 56 years.

(11) $$\begin{array}{c} \frac{v\left(x,x-1\right)}{x\left(t-1,t\right)}>\frac{v\left(x-i,x-i-1\right)}{x\left(t-i-1,t-i\right)}. \end{array}$$

According to the random method of single and double days (patients who visited the clinic on one day were included in the white light mode group, and those who visited the clinic on two days were included in the NBI mode group), they were divided into 58 cases in the white light mode group and 55 cases in the NBI mode group as shown in Table 2. There were no significant differences in gender, age, composition ratio, smoking, drinking, and other living habits between the two groups (*P* > 0.05), which were comparable.

According to the Sano classification, the telangiectasia of normal large laryngeal mucosa and proliferative lesions is not obvious, but almost all tumor lesions (adenoma or adenocarcinoma) have the expansion and thickening of the capillary network, which can be observed in NBI mode. Because of its characteristic brown capillary network structure, narrowband endoscopy is of great significance in the identification of tumor and nontumor lesions. Combining NBI with magnifying endoscopy, the accuracy rate of distinguishing neoplastic and nonneoplastic lesions in large laryngeal diseases according to the presence or absence of brown vascular network is as high as 93.4%.

## 5. Application and Analysis of Postoperative Examination Model for Laryngeal Malignant Tumor Based on Narrowband Imaging Resolution Enhancement Technology

### 5.1. Image Resolution Extraction in Different Modes

A total of 33 lesions in 30 LST patients with different imaging resolutions were selected, and the Kudo duct opening classification (Kudo classification) and the Sano mucosal surface capillary classification (Sano classification) were used in normal white light mode and NBI mode, respectively, to be diagnosed with the nature of the lesion and then undergo endoscopic resection and record the patient's gender, age, clinical manifestations, lesion location, lesion size, morphological type, pathological type, endoscopic treatment methods, and complications and other data. Statistical analysis was performed.

(12) $$\begin{array}{c} M\left\{\begin{array}{c} i\in \text{node}\left(\text{case}\right)\\ j\in \text{node}\left(\text{line}\right) \end{array}\right)=\left\{\begin{array}{c} x\in \text{node}\left(i\left(x\right),j\left(x\right)\right)\\ y\in \text{node}\left(i\left(y\right),j\left(y\right)\right) \end{array}\right\}. \end{array}$$

The biopsy detection rates of laryngeal malignant lesions in the white light mode group and the NBI mode group were calculated, respectively (malignant lesion biopsy detection rate % = the number of cases with malignant lesions found in biopsy/the number of cases with surgical resection histopathological results of malignant lesions (100%)), and correct detection rate (correct detection rate % = number of cases with consistent histopathological results between biopsy and surgical resection/total number of cases (100%)). The chi-square test was used to compare the rates, and *P* < 0.05 was considered statistically significant.

Narrowband imaging and magnifying laryngoscopy were used to observe the morphological changes of laryngeal fovea in the diagnosis of precancerous lesions (laryngealization, mild to moderate dysplasia). The detection rate was 42.8% (66/154).  Figure 6 shows the diagnosis of severe dysplasia and early laryngeal cancer. The sensitivity was 78.6%, the specificity was 95.7%, and the coincidence rate was 94.2%; the sensitivity of microvascular morphology in the diagnosis of severe dysplasia and early laryngeal cancer was 76.9%, the specificity was 97.2%, and the coincidence rate was 95.4%.

(13) $$\begin{array}{c} \text{derta}\left(x\left(\max\right),x\left(\min\right)\right)=\left\{\begin{array}{c} x\left(\max\right)-x\left(i,j\left(t,t-1\right)\right)|t\left(i,j\right),\\ x\left(\min\right)-x\left(i,j\right)|t\left(i,j\right). \end{array}\right) \end{array}$$

The positive rates of Ang-2 in mucosal inflammation, dysplasia, and laryngeal carcinoma groups were 16.4% (9/55), 42.3% (11/26), and 68.4% (13/19), respectively, and the differences were statistically significant (*P*=0.000); the positive expression rate in laryngeal cancer group was significantly higher than that in mucosal inflammation group (*P*=0.000); there was no difference in expression with dysplasia group (*P*=0.107).

### 5.2. Simulation Realization of Postoperative Examination Model for Laryngeal Malignant Tumor

Among the 58 patients in the white light pattern group, the histopathological results of the biopsy tissue examined for laryngeal malignant tumors after surgery were malignant lesions in 32 cases, including 29 cases of squamous cell carcinoma and 3 cases of carcinoma in situ; 26 cases of nonmalignant lesions, including 9 cases of necrotic tissue, 6 cases of simple hyperplasia, 7 cases of papilloma, 3 cases of vocal cord polyps, and 1 case of amyloidosis. Combined with narrowband imaging technology, we can observe whether the surface structure of gastric mucosa is regular, whether the arrangement of gastric pits is regular, and the morphological characteristics of mucosal vascular network, so as to identify benign and malignant lesions and predict the degree and stage of malignancy.

The histopathological results of surgically resected tissues in the white light pattern group were malignant lesions in 45 cases, including 38 cases of squamous cell carcinoma and 7 cases of carcinoma in situ; 13 cases of nonmalignant lesions, including 2 cases of simple hyperplasia and 7 cases of papilloma, 3 cases of vocal cord polyps, and 1 case of amyloidosis. Among the 55 patients in the NBI model group, the histopathological results of biopsy tissue were malignant lesions in 42 cases, including 36 cases of squamous cell carcinoma and 6 cases of carcinoma in situ; 13 cases of nonmalignant lesions, including 3 cases of simple hyperplasia.

(14) $$\begin{array}{c} \left(\exists f\left(x,t\right)\in T\left(i=1,j=0\right)\right)\cap T\left(i=x\left(t\right),j=x\left(t\right)-1\right)=\mathrm{mod}\text{ fiction}\left(x,y\right). \end{array}$$

There were 6 cases of papilloma and 4 cases of vocal cord polyps. In the NBI model group, the histopathological results of surgically resected tissues were malignant lesions in 44 cases, including 36 cases of squamous cell carcinoma and 8 cases of carcinoma in situ; 11 cases of nonmalignant lesions, including 1 case of simple hyperplasia, 6 cases of papilloma, and 4 cases of vocal cord polyps.

In the comparison of the accuracy of the normal white light mode and the NBI mode to diagnose the nature of the lesions, according to the classification criteria shown in Figure 7, cases of tumor lesions were to be diagnosed in the normal white light mode, the accuracy rate was 69.70%, and the tumor was to be diagnosed in the NBI mode. There were 31 cases of sexual lesions, with an accuracy rate of 93.94%. The NBI model had a higher accuracy rate for the proposed diagnosis of the nature of the lesions under the Kudo classification criteria. Using tissue microarray to study the expression of COX-2 in gastric cancer, the results showed that the positive rate of COX-2 in gastric cancer was 87.36%, and the expression rate of COX-2 in papillary adenocarcinoma and mucinous adenocarcinoma was 100%. The expression rate in normal gastric tissue was 59.0%. According to the Sano classification standard, 21 cases of neoplastic lesions were to be diagnosed in the ordinary white light mode, with an accuracy rate of 63.63%, and 29 cases of tumor lesions were to be diagnosed in the NBI mode, with an accuracy rate of 87.88%. The quasi-diagnostic accuracy of the properties is higher.

### 5.3. Example Application and Analysis

Laryngeal malignant tumor surgical instruments were as follows: Olympus CV-260SL image processing device (equipped with high-quality HDTV images and NBI function), Olympus CLV-260SL endoscope cold light source, Olympus CF-H260AI variable hardness electronic knot laryngoscope (equipped with compatible high-quality CCD photocoupler for HDTV images), ERBE 200S high-frequency electric cutting device, ERBE APC2 argon ion coagulator, Olympus NM-200U-0423 disposable submucosal injection needle, Olympus complete set of disposable electric snares 5U-1, SD-6U-1, etc., Olympus HX-110QR and HX-110UR clip device bodies, HX-20U-1 pushers, Olympus complete set of metal titanium clips (including HX-610-135L and HX-600-090, HX-610-135), MTW-GPS-21-15-230 polypectomy device, MTW-REF0910718212 injection needle for endoscopy, OlympusSZX9-31 solid microscope, etc.

In the NBI pattern group in Figure 8, the mucosal morphology and the superficial mucosal microvascular morphology of the same lesion in two different patterns were compared, and combined with the histopathological results, it was found that the histopathological results of surgically resected tissue were malignant lesions. Under the NBI microscope, the IPCL is generally abnormally enlarged, elongated, twisted, enlarged in diameter, and uneven in shape. Some are solid or hollow tan spots. If the spots are obvious and the distribution is particularly irregular, the possibility of malignancy is high. Others appear to be cord-like, twisted, and messy out of shape. In some malignant lesions, the IPCL structure has disappeared and is replaced by tumor neovascularization, with disordered and irregular distribution, uneven density, and different shapes. However, the morphological changes of mucosal microvessels in the malignant lesions of Figure 9 were not as clear in the white light mode as in the NBI mode. Compared with NBI endoscopy, the coincidence rate of EUS combined with NBI examination was significantly different from that of NBI staining endoscopy (58.33%) (*P*=0.000 < 0.05).

The histopathological results of the surgically removed tissue are simple hyperplasia because the surface of the lesion is mostly keratinized epithelium or hyperplastic squamous epithelium. In both white light mode and NBI mode, the lesion is covered by white pseudomembrane. NBI is not expressed or little expressed in various normal tissues but often overexpressed in malignant tumor tissues and acts on tumor cells by autocrine or paracrine, which is related to the metastasis, prognosis, and recurrence of various tumors. NBI mode. There were also no abnormal blood vessels. Histopathological findings of surgically resected tissue were papilloma lesions, which in NBI mode showed mild expansion of IPCL as small, sparsely arranged brown spots, while in white light mode, only gross lesions were visible. Morphology, benign, and malignant lesions can only be judged based on the clinical experience of clinicians and cannot be accurately differentiated from malignant lesions. The histopathological findings of surgically resected tissue were polyp lesions, which showed no visible IPCL on the mucosal surface in NBI mode, and only oblique vessels and dendritic vessels could be seen, similar to normal mucosa.

## 6. Conclusion

The narrowband imaging endoscope used in this paper uses its own special optical effects, combined with the biological characteristics of throat tumors, to clearly distinguish the general morphology of malignant throat lesions and the morphology of superficial mucosal microvessels from normal tissue compared with traditional endoscopy. By identifying abnormal IPCL, finding the location of malignant lesions and determining the location of biopsy tissue, the biopsy detection rate, and correct detection rate of malignant lesions of the larynx can be significantly improved, which plays a role in targeting biopsy and reduces missed diagnosis and misdiagnosis and has high clinical value. The completeness of EMR resection, the degree of tumor differentiation of the lesions, and the depth of tumor infiltration are directly related to the local recurrence after treatment, and incomplete resection is a risk factor for poor prognosis of straight laryngeal tumors. Therefore, LST patients undergoing EMR treatment should undergo standardized endoscopic followup, especially at least one nodular laryngoscopy within six months of receiving treatment. Compared with EMR, the operation time of ESD is significantly longer, the technical difficulty is more difficult, and it is more likely to cause serious complications; in addition, it has higher requirements for endoscopes and auxiliary devices, and at the same time, endoscopists are required to undergo strict technical training to reduce the operation risk and reduce the risk of operation with higher economic costs. In the process of tumor angiogenesis, NBI can not only induce angiogenesis but also facilitate tumor cells to shed into blood vessels or spread to adjacent tissues. At present, there is a lack of unified operating norms and guidelines for ESD for the treatment of LST lesions in the laryngo and larynx, and the treatment effect of LST lesions still needs to be confirmed by evidence-based medical research.

## Figures and Tables

**Figure 1:** Histogram of narrowband imaging preference assessment.

**Figure 2:** Resolution digital enhancement process.

**Figure 3:** Distribution of lesions in the larynx under the two modes of NBI.

**Figure 4:** Narrowband imaging resolution data distribution.

**Figure 5:** Distribution of postoperative recovery rate for laryngeal lesions under NBI.

**Figure 6:** Comparison of imaging resolutions in different modes.

**Figure 7:** Distribution of the lesion rate of laryngeal malignant tumor after operation.

**Figure 8:** Postoperative examination of laryngeal malignant tumor under narrowband imaging.

**Figure 9:** Distribution of histopathological results in NBI mode.

**Table 1:** Pathological statistics of laryngeal malignant tumors.

Homogeneous particles	Age/years	The average diameter/mm	Patient example ratio
10	32.078	60.557	46/100
20	48.341	46.237	52/100
30	39.401	52.648	11/100
40	46.608	2.258	76/100
50	44.537	76.900	10/100
60	28.231	10.942	48/100
70	27.410	48.931	42/100

**Table 2:** Histological results of laryngeal malignant tumors.

Histological number	NBI events	Composition ratio	Laryngeal malignant	Significant difference
100	Normal large	0.113	Magnifying endoscopy	0.213
110	Normal large	0.121	Magnifying endoscopy	0.742
120	Normal large	0.004	The capillary network	0.338
130	Proliferative lesions	0.219	The capillary network	0.086
140	Proliferative lesions	0.661	Nonneoplastic lesions	0.525
150	Proliferative lesions	0.318	Nonneoplastic lesions	0.437

## Data Availability

The data used to support the findings of this study are available from the corresponding author upon request.
